RETRACTED

# Machine English Translation Evaluation System Based on BP Neural Network Algorithm

**DOI:** 10.1155/2022/4974579

**Published:** 2022-09-21

**Authors:** Yanlin Han, Shaoxiu Meng

**Affiliations:** ^1^Shijiazhuang Information Engineering Vocational College, Shijiazhuang, China; ^2^School of Foreign Languages, Zhangjiakou University, Zhangjiakou, China

## Abstract

In order to solve the problems of machine translation efficiency and translation quality, this paper proposes an English translation evaluation system based on the BP neural network algorithm. This method provides users with a more intelligent machine translation service experience. With the help of the BP neural network algorithm, taking English online translation as the research object, Google's translation quality is the best, with an error frequency of only 167, while Baidu translation and iFLYTEK translation in China have a high error rate of 266 and 301, respectively, which is much higher than Google translation. A model of machine translation evaluation based on the neural network algorithm is proposed to better solve the disadvantages of traditional English machine translation. The results show that the machine translation system based on the neural network algorithm can further optimize the problems existing in machine translation, such as insufficient use of information and large scale of model parameters, and further improve the performance of neural network machine translation.

## 1. Introduction

The emergence and development of the network have changed the operation mode of many industries to a great extent. Of course, the biggest feature of the network is that it shortens the communication distance between people and directly breaks the distance barrier in traditional communication. However, with the support of this technology, language barriers always exist. In particular, with the in-depth development of economic globalization and integration, international exchanges are becoming more and more frequent. Business exchanges, personal exchanges, government exchanges between countries, and international academic exchanges all need the support of high-quality language translation systems. English is still the main way of international cooperation and communication, so the efficiency and quality of English machine translation are directly related to the effectiveness of international communication. Therefore, this paper proposes a machine translation evaluation system model based on the neural network algorithm to better solve the disadvantages of English machine translation, such as insufficient use of information and large-scale model parameters.

## 2. Related Works

Ma et al. said that with the rapid development of modern science and technology, international contacts have become more frequent and convenient, and exchanges between different languages have become more frequent. As an important way to break through language communication barriers, translation plays an increasingly important role in people's daily life [1]. Zhang et al. said that the traditional translation method is human translation, which relies on people who know both the source language and the target language to carry out the translation work. However, although such a translation method can obtain high-quality translation results, it has a long translation cycle and requires a lot of human and material resources. It cannot be frequently applied to people's daily lives and widely meet various translation needs [2]. Chen and Huang said that people began to focus on the use of computers to automatically translate different languages and texts, so as to achieve the goal of efficiently solving cross-language communication difficulties. Machine translation came into being [3].

RETRACTED

Jiang and Wang said that the new upsurge of machine translation in the 1970s was determined by actual needs [4]. Huang et al. said that with the development of science and technology, the exchange of national scientific and technological information is becoming more and more frequent, and the language barriers between countries are becoming more and more intense [5]. At that time, any document of the European community had to be translated into six languages; Canada adopts a bilingual system, and its government documents must be translated into English and French; and due to the development of foreign trade, Japan needs a large number of exports. The translation task of export product manuals and various instant news is very huge. Liang and Li said that the traditional labor translation practice is far from meeting the demand, and there is an urgent need for computers engaged in translation [6]. Chen et al. said that the new upsurge of machine translation in the 1970s was also related to automatic retrieval and artificial intelligence [7]. Xu et al. said that with the progress of modern science and technology, machine translation in the 1970s was no longer a topic of natural language processing [8]. Sreelekha et al. said that to establish various information retrieval systems, it is necessary to automatically index documents and even use computers to process natural languages. It is necessary to solve the problem of automatic analysis of natural language texts, which is closely related to machine translation [9].

Lalrempuii et al.said that, in the first stage of the establishment of machine translation in 1957, the Institute of Languages of the Chinese Academy of Sciences and the Institute of Russian-Chinese Machine Translation Computing Technology cooperated to translate nine different types of complex sentences [10]. However, due to the international situation and inherent difficulties of machine translation, the second stage of the history of Chinese-English machine translation stagnated, and little progress was made in the study of Chinese-English machine translation during this period. The third stage of machine translation, the vigorous development stage, began in 1975. Machine translation has been listed as China's “Sixth Five-Year Plan,” “Seventh Five-Year Plan,” “863,” and other major scientific research topics. Researchers have concentrated on cooperative research in multiple research institutions and ministries, and have carried out cooperative exchange projects with international research institutions. At present, Tsinghua University, Northeastern University, and other universities in China are committed to machine translation research, as shown in Figure 1.

RETRACTED

## 3. Method

Compared with the traditional rule-based machine translation model, although statistical machine translation has many advantages, there are still many challenges. For example, statistical machine translation requires many artificial features, but these features cannot cover all the language rules; statistical machine translation is difficult to take advantage of the global features; and statistical machine translation relies on many preprocessing tasks, such as word alignment and rule extraction. If syntactic features are defined, syntactic analysis is required first. This pipelined architecture will make errors in every link, errors will gradually affect the subsequent processing work, and the impact on the translation effect will be greater and greater. Facing the challenge of statistical machine translation, a better solution is to use deep learning to build models. Machine translation based on the deep learning framework model can be roughly divided into two categories. One category is still based on the statistical machine translation system and uses deep learning to improve the key modules, such as the language model, translation model, and sequencing model. [11].

Another method of the machine translation model using machine learning is to use a neural network to directly map the source language sequence into the target language sequence instead of a statistical machine translation system as the framework, word alignment, and other preprocessing and artificial design features.

To transform the problem of natural language processing into a problem of machine learning, the first step must be to find a way to mathematicize these symbols [12, 13]. In natural language processing, the simplest word representation is one-hot representation. This method represents each word as a very long vector, the word representation. Most points are 0, and only one dimension has a value of 1, which represents the current word. The word vector in deep learning is a low-dimensional real vector. The word vector will make some words closer, such as related words or similar words. This distance is usually defined according to the European distance and the cosine of the included angle. Word vector can not only avoid the disaster of dimension, but also because the distance between similar words or related words is very small, the model constructed by the word vector itself has flatness [14].

RETRACTED

Word patterns play an important role in making natural words. Practically speaking, word patterns measure the validity of sentences or use temporal expressions to measure the validity of people. It is widely used in many natural language processing tasks, such as speech recognition, part of speech tagging, machine translation, and so on.

We suppose that the word sequence w consists of *i* words, as shown in the following formula (1):

(1) $$\begin{array}{c} \omega =\omega_{1},\omega_{1},\cdots ,\omega_{t}. \end{array}$$

Then, the generation probability of word sequence is shown in the following formula (2):

(2) $$\begin{array}{c} \begin{array}{c} P\left(\omega \right)=P\left(\omega_{1},\omega_{2},...,\omega_{t}\right)\\ =P\left(\omega_{1}\right)P\left(\left.\omega_{2}\right|\omega_{1}\right)P\left(\left.\omega_{3}\right|\omega_{1},\omega_{2}\right)...P\left(\left.\omega_{t}\right|\omega_{1},...,\omega_{t-1}\right). \end{array} \end{array}$$

If the Markov assumption is used, that is, the probability of the current word is only related to the previous word, the model is simplified as shown in the following formula (3):

(3) $$\begin{array}{c} P\left(\omega \right)=P\left(\omega_{1}\right)P\left(\left.\omega_{2}\right|\omega_{1}\right)P\left(\left.\omega_{3}\right|\omega_{2}\right)\cdots P\left(\left.\omega_{t}\right|\omega_{t-1}\right)\text{.} \end{array}$$

The above is the n-gram binary grammar model. If the probability of extending it to the current word is related to the previous n-1 words, the n-gram binary grammar model is formed, as shown in the following formula (4):

(4) $$\begin{array}{c} P\left(\left.\omega_{t}\right|\omega_{1},\cdots \text{,}\right)=P\left(\left.\omega_{t}\right|\omega_{t-n+1}^{t-1}\right)\text{.} \end{array}$$

The N-gram model is relatively simple. At present, the most commonly used language model is the n-gram grammar model. However, due to the lack of n-gram words in the training corpus, which is very common, it is easy to cause data sparsity, so some smoothing algorithms need to be used in the model. Common smoothing algorithms include additive smoothing algorithm, Kneser–Ney smoothing algorithm, Katz smoothing algorithm, Jelinek–Mercer smoothing algorithm, etc. As the context length increases, the number of n-gram grammars will increase exponentially, which will prevent the model from effectively capturing long context types. This is the biggest drawback of the N-gram model. Therefore, Bengio et al. came up with the idea of applying the neural network to the language model and overcome the exponential increase in parameters by sharing parameters between similar I data [15].

RETRACTED

Learning the joint probability function of word sequences in a language is a goal of statistical language models. However, due to the disaster of data dimension, the learning of language models becomes difficult, especially when learning the joint distribution of many discrete random variables or the discrete distribution in data mining.

Dimensionality destruction should be avoided by studying word representations of words. This classification allows each sentence to be modeled on an exponential number of sentences with similar semantics. The model can learn the probability of distributed representation of each word and the distributed representation of word sequence at the same time.

The statistical language model can be expressed in the form of conditional probability multiplication, as shown in the following formula (5):

(5) $$\begin{array}{c} \hat{P}\left(\omega_{1}^{T}\right)=\overset{T}{\underset{1}{\prod }}\hat{P}\left(\frac{\omega_{t}}{\omega_{1}^{t-1}}\right), \end{array}$$

where *ω*_*t*_ is the t-th word, as shown in the following formula (6):

(6) $$\begin{array}{c} \omega_{i}^{j}=\left(\omega_{i},\omega_{i+1},\cdots ,\omega_{j-1},\omega_{j}\right). \end{array}$$

The above formula represents a string of words. As a matter of fact, we know that the words close to each other in the word sequence are statistically more dependent. Therefore, using the N-ary grammar model, we can get the following formula (7):

(7) $$\begin{array}{c} \hat{P}\left(\left.\frac{\omega_{t}}{\omega_{1}^{t-1}}\right|\right)\approx \hat{P}\left(\frac{\omega_{t}}{\omega_{t-n+1}^{t-1}}\right). \end{array}$$

Here, only the combinations of continuous words that appear frequently enough in the training corpus are considered.

The neural probabilistic language model uses the neural network model to estimate P(*ω*_*t*_/*ω*_*t*−*n*+1_^*t*−1^). The training set of the model is a sequence, as shown in Figure 2.

RETRACTED

Figure C from element I in V to the actual vector (see Figure 2) represents the representation of each word in the word and its corresponding attribute. In fact, C represents a matrix of |*V*| × *m*. If G is used to represent the probability function of a word, function *g* represents the conditional probability distribution from the input order of the feature vector of the word in the context to the next word in word *v*. Therefore, combining these two steps can obtain the result as shown in formulas (8) and (9).

(8) $$\begin{array}{c} C\left(i\right)\in R^{m}, \end{array}$$

(9) $$\begin{array}{c} f\left(i,\omega_{t-1},\cdots ,i,\omega_{t-n+1}\right)=g\left(i,C\left(\omega_{t-1}\right),\cdots ,C\left(\omega \left(t-n+1\right)\right)\right)\text{.} \end{array}$$

Therefore, function *f* is a composite of mapping C and *g*, and the parameter of mapping C is the eigenvector itself, which is represented by a |*V*| × *m* matrix, where the line I of the matrix is the eigenvector of word *i*. Function *g* can be realized through a feedforward neural network, recursive neural network, or other parameter functions. Assuming its parameter is *ω*, all the parameter sets are as shown in the following formula (10):

(10) $$\begin{array}{c} \theta =\left(C,\omega \right)\text{.} \end{array}$$

The training is realized by finding the *θ* with the largest penalty logarithmic function in the stem training language library, as shown in the following formula (11):

(11) $$\begin{array}{c} L=\frac{1}{T}\underset{t}{\sum }\log\;f\left(\omega_{t},\omega_{t-1},...,\omega_{t-n+1}\right)+R\left(\theta \right), \end{array}$$

where *R*(*θ*) is a normal female operator *f*. In this paper, *R* is a weighted penalty function, which acts on matrix C in the neural network.

In the later experiments, in addition to the feature vector mapping layer, there is a hidden layer in the neural network structure, which is directly connected to the output layer through the feature vector mapping layer. Therefore, there are two hidden layers in the model: the C layer that shares linguistic features and the hyperbolic tangent hidden process. In fact, the neural network also has a set of algorithms to ensure that its results are positive, and the result of each result is 1. Its calculation formula is as shown in the following formula (12):

(12) $$\begin{array}{c} \hat{P}\left(\left.\omega_{t}\right|\omega_{t-1},...,\omega_{t-n+1}\right)=\frac{e^{y_{wt}}}{\sum e_{i}^{y_{i}}}, \end{array}$$

where *y*_*i*_ is the irregular logarithmic probability of the output word I, which is calculated by the formula composed of parameters *b*, *W*, *U*, *d,* and *H*, as shown in the following formula (13):

(13) $$\begin{array}{c} y=b+Wx+U\;\tanh\;\left(d+Hx\right), \end{array}$$

where *W* can be 0, which means that there is no direct connection between the feature vector layer and the output layer, and *x* is the vector of the word feature layer and the connection of the input word feature vector from matrix C, as shown in the following formula (14):

(14) $$\begin{array}{c} x=\left(C\left(\omega_{t-1}\right),C\left(\omega_{t-2}\right),...,C\left(\omega_{t-n+1}\right)\right). \end{array}$$

Therefore, the parameter set is as shown in the following formula (15):

(15) $$\begin{array}{c} \theta =\left(b,d,W,U,H,C\right). \end{array}$$

The number of free parameters is as shown in the following formula (16):

(16) $$\begin{array}{c} \left|V\right|\left(1+nm+h\right)+h\left(1+\left(n-1\right)m\right). \end{array}$$

The number of parameters that play a leading role is |*V*|(*nm*+*h*), where *h* refers to the number of neurons in the hidden layer.

RETRACTED

## 4. Experiment and Analysis

The transformer system and ConvS2S system are the existing advanced NMT systems. They rely on the self-attention mechanism and CNN for sequence modeling, respectively. They are typical representatives of NMT systems. Among them, encoder and decoder are stacked by multilayer networks, which is a common feature between them [16].

Transformer is modeled by the self-attention mechanism sequence, which is an important feature that distinguishes it from other machine translation systems. Its framework is shown in Figure 3. Transformer has become the current mainstream framework because of its outstanding performance. It uses the source-side self-attention mechanism and the target-side self-attention mechanism to model the source language sequence, as shown in the following formulas (17) and (18):

(17) $$\begin{array}{c} X=\left(x_{1},x_{2},...,x_{m}\right). \end{array}$$

Target language sequence is as follows:

(18) $$\begin{array}{c} Y=\left(y_{1},y_{2},...,y_{m}\right). \end{array}$$

The transformer system encoder is stacked by N layers of networks, and each layer is composed of a self-attention mechanism sublayer and a feedforward neural network sublayer, as shown in Figure 3.

We obtain the corresponding information representation. The self-attention mechanism is used to calculate the weight of each word in a sentence and all words in the sentence, so as to obtain the internal correlation between words [17, 18].

The transformer system encoder consists of n-layer networks, and each layer consists of a self-listening mechanism sublayer and a feedforward neural network sub-layer. The decoders are also stacked by network layers, which have one more attention sublayer than the encoder. The output of each layer is processed by layer normalization, which helps to accelerate the model training of the deep network. Residual connection is used between sublayers to avoid the problem that it is difficult to transfer gradients in multilayer networks [19].

RETRACTED

This article selects the keynote speech at the opening ceremony of the Boao Forum for Asia Annual Conference 2018 as the review object. There are 5652 words in the text, 3821 words in Google translation, 3805 words in Baidu translation, 3614 words in iFLYTEK translation, and 3777 words in translation. The author compares the definitions of mustard song, listening degree, and iFLYTEK with the translation file of more than 20,000 words word by word [20, 21]. Before comparing the whole UI, the author first randomly takes iFLYTEK as the first analysis object to find out the unsuccessful translation of the target language and mark all errors from beginning to end. According to the three levels described by karljames—ontology errors, text errors and text errors, and various subcategories, corresponding additions and deletions are made according to the characteristics of machine translation. Finally, four first-class types (including “other errors”), ten second-class types, and several third-class, fourth-class, and fifth-class types are determined. Subsequently, on the basis of the error types, we identified the errors in the translations of Google and Baidu. In general, we conducted three repeated error screenings on the translations of the three machine translation companies, and constantly added, deleted, and adjusted the error types in the process, so as to ensure the quality of the comparative study of the translations.

The ultimate goal of error classification in this paper is to propose error correction strategies for machine translation and ultimately improve the translation quality of machine translation. Therefore, “understanding errors” is one of the key objects of error classification. All noun errors with substantive information are classified as “connotative errors” or “information omission,” but not as “noun errors” or “noun omission” [22]. In the process of error marking, in order to avoid repetition and make the analysis results have no guiding significance, this paper marks a specific error repeated in an article as “1.” For example, in iFLYTEK translation, the term “annual meeting” is translated into “annual meeting” rather than the correct “Annual Conference.” Even if it occurs many times, the term error is counted as “1,” as shown in Table 1.

Through the identification and diagnosis of errors, this paper classifies, makes quantitative statistical analysis and memory description according to the types, levels, and frequencies of errors, and puts forward corresponding correction strategies.

RETRACTED

After a comprehensive parallel sentence-by-sentence comparison and error location between the machine translation and the official translation, the author uses Excel to classify, count, and summarize the error levels and their frequencies in the machine translation. The quantitative description and qualitative evaluation of the whole and individual and the corresponding corrective strategies will be carried out, as shown in Table 2:

As shown in Table 2 and Figures 4–6, from an overall perspective, the error rate of Google, Baidu, and iFLYTEK in handling the keynote speech of the chairman at the Boao Forum for Asia in 2018 is far lower than that of the other two (44.5% lower than iFLYTEK and 37.2% lower than Baidu). From the perspective of error occurrence, errors are concentrated at the discourse level, accounting for up to half of the total error frequency, and at the discourse level, accounting for nearly 40% of the total error frequency. Second, ontology errors account for more than 10% of the total error frequency. Only iFLYTEK translation has “other errors,” and the error frequency is far lower than that of other error levels. Next, this paper will analyze the error strength with higher frequency and better guiding significance [23, 24], as shown in Figures 4–6.

From the frequency statistics of error types, the frequency of ontology errors accounts for the percentage of the total number of errors, but the error information of the opening text and segmented sentence deletion is more concentrated than other types of errors; in terms of the performance of the translator, Google Translate has the best performance. It outperforms the other two on the first line of text and error lines [25]. It can be seen that although Google's machine translation has made some achievements in Chinese recognition, Chinese recognition and sentence breaking are still the focus of machine translation researchers. In the aspect of recognition and sentence breaking, the main mistakes of machine translation lie in the following: (a) unable to correctly identify Chinese sentence structures, especially coordinate structures, partial structures, and subject-predicate structures; (b) it is unable to deal with long sentences with complex sentence structure, so it can only be literally piled up, which cannot convey any H-line effect meaning in English; (c) and broken sentences lead to too long machine translation, which makes it difficult for readers to read, as shown in Figure 7.

Semantic errors include four categories: term errors, misuses of synonyms, semantic range differences, and stylistic misuses. According to the statistical data on the frequency of error types, terminology errors rank first. However, in the field of machine translation, the severity of terminology problems is low, which can be supplemented by enhancing relevant corpus training. However, it is urgent to solve the problem of vocabulary selection [26, 27]. Vocabulary is the brick and tile of language. The choice of vocabulary is very important to the quality of translation, and it is the basic element of linking words into sentences. In terms of semantic errors, the performance of the three machine translation systems is equal, and the gap is not large, so they all need to be improved, as shown in Figure 8:

Syntactic errors are the hardest hit area of paragraph errors and the bottleneck of machine translation. For the translation of terms, researchers can also input them into the corpus for training. For the ever-changing sentences, the “dictionary” translation based entirely on the historical corpus cannot meet the needs of users for high-quality translation. Although the three machine translation systems studied in this paper have made great achievements in the automatic translation between natural languages through artificial intelligence through neural networks, some studies have pointed out that in the translation of multiple samples, the computer via network machine translation system has reduced the error by 55%–85% or more. In terms of the total frequency of errors made by machine translation systems, errors mainly occur in the misuse of sentence components and information omission (as shown in Figure 9), and all three machine translation systems output a large number of invalid sentences: from the perspective of the platform, Google Translate performs best at the syntactic level, and among the three machine translation platforms, it can reduce the burden on post-translation editors, which has certain reference significance.

RETRACTED

The problem of information omission accounts for nearly 40% of the total syntactic error rate, especially the problem of information omission of iFLYTEK. Compared with Google's omission of some information in a sentence, iFLYTEK and Kedu will miss the whole sentence of multiple sentences. According to the results of this experiment, the completion rate of machine translation is not high, and it cannot reach the level of being competent for human translation tasks in a short time. Its main role should be to reduce the burden of post-translation editors. If there is a large number of missing translations, it will increase the burden of post-translation editors.

From the above research, it can be found that for the text studied in this paper, Google's translation quality is the best, and the error frequency is only 167, while the error rate of domestic Baidu translation and iFLYTEK translation is higher, 266 and 301 respectively, which is much higher than Google translation. It proves that domestic translation software does not have advantages in Chinese-English translation of texts with Chinese characteristics but still lags behind international software. At the level of ontology errors, Baidu and Google perform poorly in the identification and sentence breaking of the original text. The frequency of errors is 20 or more. On the contrary, Google translation only occurs 10 times. Domestic software should have inherent advantages in Chinese recognition and corpus construction, but research shows that it still lags far behind Google translate in this regard, and cannot recognize and break Chinese well [28].

At the level of paragraph errors, the performance of most of the three mainstream translation systems is similar, and the frequency of errors is similar, but there are significant differences in the level of “information omission”: Google translation only has 8 information omission errors, while Baidu translation has 25, and iFLYTEK translation has 73 information omission errors, which cannot meet the standard in the first level of “faithfulness.” As mentioned above, the main advantage of neural network machine translation is that it can get smoother and more close to natural language translation, which is more fluent and readable, but it may lead to the translation being unfaithful to the original text, that is, the translation may be very smooth, but it does not match the original text well, and output a “self-created” language. The iFLYTEK translation in this paper clearly reflects this weakness. At the same time, it can be found that most of the missing information is difficult for human translators to deal with. The three machine translation systems may not have trained this kind of corpus and gradually omit it in a wide range of translation. At the level of discourse errors, the types of errors with sexual shame are comprehension errors—ambiguity and connotation. The error frequency of Google and iFLYTEK translation is 30+ and that of Baidu translation is twice as high as that of the first two, indicating that Baidu translation needs to further strengthen systematic training in the “context” and enhance the ability of machine translation to select appropriate words and sentences in the context.

Although the translator has developed to a certain extent, the current tools are not mature enough to deal with difficult sentences and understand the deep meaning of words, the corpus training is also very low, and the physical ability is insufficient, so it is difficult to achieve a more systematic and more accurate translation, a sound education; the combination of machine translation and linguistic research is not yet complete, and translation cannot be handled scientifically from the linguistic level. Many reasons have led to frequent machine translation errors.

RETRACTED

This chapter mainly makes quantitative and qualitative statistics and research on the errors of machine translation, adds the analysis of typical cases of error types with research value, and summarizes the main reasons for the limitations of machine translation at present.

## 5. Conclusions

In this paper, based on the theoretical perspective of error analysis, the author sets up an evaluation model of machine translation error analysis. Taking the keynote speech and official translation of President Xi Jinping at the Boao Forum for Asia in 2018 as the test corpus, the author compares and analyzes the translation quality of three major neural network machine translation systems: Google, Baidu, and iFLYTEK. It classifies and sorts out the types of errors made in the three levels of ontology, text, and discourse, makes quantitative and qualitative analysis, and puts forward corresponding countermeasures. In this chapter, the author will briefly summarize the findings and limitations of this study, and put forward prospects for future research.

There are few errors in machine translation at the ontology level, which reflects that machine translation has made great progress in Chinese recognition, but there is still much room for improvement. After all, the correct recognition of Chinese and punctuation is the basis for accurate translation. The recognition of “shanqinghaixiu” as “mountain and Qinghai” is a small mistake, but it deeply reflects the current recognition level of machine translation and the lack of understanding of Chinese logic. In addition, the three machine translation companies all lack reasonable recognition of the role of “stop sign.” The occurrence of stop sign in long sentences has seriously affected the sentence breaking of machine translation, resulting in serious semantic confusion and invalid stacking of words.

In the aspect of paragraph development, a large number of errors in machine translation prove that machine translation still has strict defects in word formation and sentence formation. If the translated sentences fail to conform to the English grammatical norms, machine translation will lose its original role and become a stack of words (groups). Under the semantic type, the misuse of terms, synonyms, semantic range, and style all reflect the shortcomings of word selection in machine translation. Although the general view is that the terminology problem is easy to solve and only needs to input corpus to strengthen training, the author believes that relying only on historical corpus should not be the main way of machine translation but should strengthen the predictive ability of machine translation. Taking the “community of human destiny” as an example, the translation of this important term has been analyzed and determined in detail on the internet. Whether machine translation can actively search the relevant corpus for learning and judgment, whether there is already a bilingual corpus of “XX community” in the historical corpus, and whether machine translation can predict according to the context are a topic that researchers can deepen. Under the type of syntactic errors, machine translation makes errors in the form, phrase structure, sentence components (mistranslation, redundancy, or deletion), part of speech, tense and voice, omission, and unity, and even outputs many invalid sentences. It is worth mentioning that iFLYTEK translation, which has the highest error rate, has a lot of problems of missing information and making things out of nothing. This just reflects the weakness of neural network machine translation—as mentioned in the previous literature research, the translation language obtained by neural network machine translation is closer to natural language, and its fluency can avoid “translation cavity” and facilitate people's understanding, but the fidelity of the translation is still in doubt. However, this study proves that if the training direction of neural network machine translation shifts, the translation results will be wrong (i.e., unfaithful to the original text) but very smooth. Text level is also a difficult problem for manual translators, and machine translation makes many mistakes at this level. There is a lack of logical coherence between machine translation sentences, and the handling of culture-loaded information and metaphors is also dismal. The transmission of many information is only superficial and unable to convey the real meaning of the speaker, which will also cause ambiguity. In addition, many of the same words are repeated twice in a row and the same meaning is repeatedly expressed.

RETRACTED

## Figures and Tables

**Figure 1:** Machine translation research.

**Figure 2:** Neural probabilistic language model.

**Figure 3:** Transformer benchmark system.

**Figure 4:** Total number of machine translation errors in the three companies.

**Figure 5:** Overall error frequency at all levels.

**Figure 6:** Statistical chart of three machine translation error types.

**Figure 7:** Statistical diagram of ontology errors in three machine translation errors.

**Figure 8:** Frequency of semantic errors in paragraph errors.

**Figure 9:** Frequency of syntactic errors in paragraph errors.

**Table 1:** Machine translation error types.

Level 1 error	Body error	Semantic error	Semantic cohesion	Creating somethingout of nothing
Level 2 error	Misspelling	Syntactic error	Pragmatic error	
	Punctuation	Term error	Interpretive error	
	Original text recognition andsentence-breaking errors	Misuse of synonyms	Repetitive redundancy	

Level 3 error	Case	Semantic range inequality	Conjunctions and logic	Component
	Comma, period, andquotation mark	Semantic error	Cultural load and metaphor	Punctuation
		Syntactic error	Ambiguity and connotation	

**Table 2:** Summary of error levels and frequency of each platform.

Error segmentation	Google (frequency)	Baidu (frequency)	iFLYTEK (frequency)
Misspelling	1	7	8
Punctuation	2	8	5
Original text recognition and sentence-breaking errors	10	24	20
Misuse of synonyms	1	3	7
Semantic range inequality	2	0	2
Misuse of style	2	3	5
Singular and plural number matching	0	2	1

## Data Availability

The data used and/or analyzed during the current study can be obtained from the corresponding author upon request.
